# The Practice and Application of AR Games to Assist Children's English Pronunciation Teaching

**DOI:** 10.1155/2022/3966740

**Published:** 2022-06-30

**Authors:** Liang Hu, Yuan Yuan, Qing Chen, Xiangying Kang, Yan Zhu

**Affiliations:** ^1^School of Foreign Studies, Hunan First Normal University, Changsha, 410017 Hunan Province, China; ^2^School of Foreign Languages, Hunan University of Humanities, Science and Technology, Loudi, 417000 Hunan Province, China; ^3^School of Foreign Languages, Central South University, Changsha, 410083 Hunan Province, China; ^4^School of Foreign Languages, Hunan University of Technology and Business, Changsha, 410017 Hunan Province, China

## Abstract

This paper conducts an in-depth study and analysis of the practice and application of teaching English pronunciation to children using AR (augmented reality) game assistance. The article analyzes the design of AR educational games based on the concept of learning behavior input, clarifies and determines the factors influencing students' learning behavior input in AR gamified teaching environment, and proposes the design principles of AR educational games based on learning behavior input. By analyzing the characteristics of experiential learning and AR, the model of AR-based English experiential learning activities for elementary school is established. Based on certain demand analysis, the AR software that can be used for teaching pronunciation in elementary school English classrooms was designed and developed using Unity3D and 3ds Max software. The experimental method was used to compare and apply the software in the target school, and the students of elementary school X were selected as the experimental subjects. The data were analyzed with the help of SPSS and NVivo software, and the questionnaire was used to measure the “ease of use,” “usefulness,” and “satisfaction with the software.” The questionnaire was used to measure students' acceptance of AR software in three dimensions: “ease of use,” “usefulness,” and “satisfaction with the software.”

## 1. Introduction

It is undeniable that we all like to be entertained and to play games, and so do students, and this has drawn the attention of experts in the relevant fields who have tried to introduce the mechanisms, concepts, and elements of games into classroom teaching, and educational games are the product of this research process. In the context of the information age, there are numerous attempts and researches on the application of various emerging technologies in the field of education, which bring changes and challenges to education teaching and at the same time present a trend of integration and development with the teaching of various subjects [1]. With the rapid development of information technology in recent years, the Internet infrastructure has been increasingly improved and the scale of Internet users has grown at a high speed. The Internet has deeply influenced children since they started to receive an education. They no longer stick to the small family around them but look at the whole world with curiosity. They are the most easily seduced individuals in the face of anything new and emerging. Growing up under the shroud of the Internet, children no longer feel new to traditional games. In terms of age structure, the younger the Internet users are, the greater the proportion is [2]. Therefore, it is the colorful and modern multimedia games that are popular among children. In the wave of new curriculum reform, student-centered “game-based teaching” has strongly influenced the traditional teaching model. The existing teaching strategies can no longer meet the goals of elementary school English classroom teaching. In the AR environment, learners can independently choose the communication scene, object, and difficulty, etc., and practice repeatedly until they are proficient. In this environment, the emotional needs of the learners are met, and the anxiety of the learners is effectively reduced. The multimedia gamification strategy is in line with the new concept advocated in the new curriculum and highlights learning through perception, experience, practice, participation, and cooperation, as well as the integration of effective strategies in the learning process to develop good learning attitudes and promote the ability of integrated use.

Augmented reality (AR), as an emerging technology, has received a lot of attention from various fields of society. And its features such as immersiveness and interactivity make it popular in the field of education at the same time. In the long history of technology-assisted education and teaching, the emergence of new technologies often brings new opportunities to education and teaching, and augmented reality is no exception. Traditional computer-assisted teaching has gradually revealed its drawbacks in the wave of new technologies, such as still mainly in the form of teacher explanation, lack of immersion, and weak interactivity. Augmented reality technology can effectively compensate for these disadvantages [3]. The interactive technical features of augmented reality technology can provide learners with a virtual learning environment that is contagious and closer to the real situation. Introducing augmented reality technology as a new form of media into education teaching, its application value has become a research hotspot in the field of education. In short, the application of augmented reality technology in the field of education provides a new way and practice area for technical support of education teaching. In general, the threshold is defined as 20 pixels. When the distance between the center point of the target position and the actual target position point estimated by the algorithm is less than the threshold pixel point, the tracking fails.

The integration of AR technology and educational games is the trend, which will greatly expand the application field of educational games. In addition, the popularity and development of smart mobile devices provide a convenient platform for the application of AR educational games in education teaching, and AR educational games will usher in a new wave of educational technology research [4]. It can increase students' experience in the learning process and cultivate their interest in learning. Therefore, AR technology-based experiential learning activities meet the requirements of the new curriculum for elementary school English teaching and have great potential for application. Based on the above background, this paper explores the practice and application of AR games to assist children's English pronunciation teaching and explores how to design the interaction of children's English pronunciation learning to increase children's attraction to the learning content and improve their English pronunciation level with strong practical significance [5].

## 2. Related Works

The gaming industry is huge, generating billions of dollars each year while using games in a way that helps students easily grasp classroom concepts and improve collaboration, communication, creativity, and imagination. AR games allow players to create virtual characters or objects and connect them to the real world in a specific location [6]. The combination of AR games and education has huge promise and can be easily applied to a range of subjects, including archaeology, history, biology, and geography. An AR video game called Alien Contact is being used in the basic education level curriculum to increase student interest and engagement [7]. The goal of the game is to discover why aliens came to Earth and landed in a specific area. Students are organized into teams before the game, with each student taking on a different role using a handheld device to complete questions by collecting evidence and instructing students to form hypotheses, and the game requires the use of limited math, science, and language arts skills. Gu et al. of East China Normal University published an augmented reality English word game for elementary school students in China's Education Through Technology, in which learners select virtual 3D characters through augmented reality and the characters are generated in the real environment where the learners are located and interact with the characters through situational quizzes. In this game, learners select virtual 3D characters in the form of augmented reality [8]. Hsu analyzed the immersion experience, perceived usefulness, and the relationship between immersion experience, perceived usefulness, and play behavior intention of adolescents aged 9-12 years old who participated in an educational game, using an RPG-like educational game “Learn and Play” as a research environment and established a conceptual model of factors influencing play behavior intention of educational game participants [9]. In the UBICARE project, Homer et al. designed and built a system to facilitate inpatient treatment and designed and implemented various learning services using a gamification approach [10].

In preschool education, the role of AR technology is to stimulate students' interest in learning. By observing the learning performance of preschoolers, we can find that they are not too fond of the boring book knowledge, but like the lively and interesting games [11]. Therefore, to stimulate preschoolers' learning interest and enhance their learning effect, there are many AR e-books on the market, mostly presenting relevant teaching content in the form of 3D models and animations, and transferring the knowledge contents to students while stimulating their learning interest. For example, Bakhsh developed a set of learning materials to help students learn Chinese phonetic symbols and applied them in a specific kindergarten classroom to explore whether they could facilitate the learning of preschoolers compared with traditional paper-based teaching resources [12]. Liu applied augmented reality to their students' learning of fables, providing them with 3D models, audio, and related interactive props, and found that their students' interest in learning was greatly enhanced [13].

In the formal classroom, the main form is “mobile device + APP.” In the formal classroom, the main forms of AR-assisted teaching are mobile devices (cell phones, iPods, etc.) and APPs, which indicates that these teaching resources are convenient and provide the possibility of promoting their use in the future. According to related research, AR technology has advantages over traditional teaching media in teaching knowledge of spatial structure, language learning, and understanding semantics. However, in language learning, most AR educational applications use AR technology as a tool to assist students in learning English words and do not apply AR technology to the teaching process of language learning in a real sense. To sum up, the research on the educational applications of virtual reality and augmented reality is still in the exploration stage at home and abroad, and although many researchers have conducted relevant research on the application of augmented reality technology in various educational stages and have obtained certain research results, there are still many problems that need to be solved [14]. Relevant researchers should increase the research on the application of AR technology in the formal English classroom and make the best possible use of the advantages of AR technology to help students learn English words more easily and effectively, improve their oral communication skills and thus stimulate their interest in learning English.

## 3. Design of an AR Game-Aided Model for Teaching English Pronunciation to Children

Augmented reality technology incorporates a variety of modern technologies such as intelligent display, tracking registration, and human-computer interaction. The function of intelligent display technology is mainly to realize the superimposition of virtual information in the real world, and its main device terminals are head-mounted displays, computers, and smartphones. Among them, the head-mounted display gives the best experience to users because it is designed according to the structure of the human body, but its application is small because of its high production difficulty [15]. The cell phone, which is already in popular use worldwide, has become the best choice for applying augmented reality technology. Registration tracking technology can realize the position correspondence between real things and virtual information, and if the position of real things has changed, the technology can also be repositioned to realize the superposition of virtual information. Human-computer interaction technology is mainly for connecting system input and output, and it is mainly divided into strong interaction and weak interaction. Strong interaction gives users a better experience but is more difficult to implement, while weak interaction gives users a worse experience but is less difficult to implement. Traditional junior high school English teaching often presents teaching content in stylized language. In communication, the information and memory stored by students are often stolen in exchange for a smooth communication process.

A total of 80 students, 50% of whom were boys (40) and 50% of whom were girls (40), from two-second grade classes in a general type of elementary school in X city were selected as subjects, and two English teachers participated in the experiment. The subjects were between the ages of 7 and 9 years old, with Chinese as their native language and English as their second language. All subjects were divided into a control class and an experimental class by the teachers of each class according to the learners' previous performance. The degree of students' exposure to AR devices in the two groups of classes was normally distributed, and the difference in the degree of students' knowledge between the two classes was not significant. Meanwhile, the percentage of students with more than general exposure to AR devices in the control class reached 65.7%, which can be considered favorable for the teaching of AR educational game implementation.

Game design is the basis for game development and implementation, and a good game design should be interesting, easy to use, and attractive. The design of educational games should include two parts: instructional design and game element design. Game element design is the core part of AR educational game design, which should include the following key categories: game interface design, game scene design, game rule design, and game main function design. Based on the analysis of game requirements, this section constructs a specific design framework for AR educational games based on the design principles of AR educational games based on learning behavior input and analyzes the specific design of the AR educational game “Knowing Phonetic Friends” for elementary school science, to provide a basis for the subsequent development and implementation of the game. The design framework of the AR educational game is shown in Figure 1.

This phenomenon can be attributed to the “game transfer phenomenon” (“Game Transfer Phenomenon”) in psychology. After the game, players will recall the previous game music and game scenes in their brains and cannot be separated from the game for a long time. SIFT feature descriptors represent the local features of an image, and the descriptors are unique and multiquantitative, which enables them to maintain strong discriminative ability and better robustness in a massive database. SIFT describes the detected feature points by a set of 128-dimensional feature vectors, and the information contained in the feature vectors includes the feature points and their surrounding pixel points, in which this joint information can improve the fault tolerance and noise immunity of the descriptors. To achieve rotational invariance of the image, SIFT defines a principal direction for the feature points by the statistical histogram, which is aligned with the principal direction of the feature points by the coordinate axis rotation operation during feature point matching.

(1) $$\begin{array}{c} \left\{\begin{array}{c} x=\cos\theta +\sin\theta ,\\ y=\sin\theta -\cot\theta , \end{array}\right. \end{array}$$

(2) $$\begin{array}{c} X_{c}={rX}_{m}=\left[\begin{array}{cc} t & 0\\ 1 & r \end{array}\right]X_{m}. \end{array}$$

To make the feature point matching algorithm usable on mobile devices and in real time, it is required that the feature descriptors are computationally small and fast. BRIEF is an algorithm that generates binarized descriptors, which not only has a low extraction cost but also matching can be done using simple Hamming distances and using the dissimilarity operation between bits. Therefore, the time cost and space cost are both low, so it is suitable for performance-constrained mobile devices. However, the BRIEF descriptor is not rotation invariant and the descriptor does not exploit any hardware features of the mobile device. Therefore, in this paper, we propose a new binary feature descriptor BRIEF, which introduces the rotation of mobile device inertial sensors, in conjunction with the hardware characteristics of mobile devices parameter to be rotationally invariant.

(3) $$\begin{array}{c} f_{n}\left(p\right)=\overset{T}{\underset{1\leq i\leq n}{\sum }}\lambda \left(y_{i},x_{i}\right), \end{array}$$

(4) $$\begin{array}{c} f_{n}=\underset{1\leq i\leq n}{\sum }2^{i}\lambda . \end{array}$$

Unity 3D is a fully integrated professional design and development engine developed by Unity Technologies, Inc. for creating interactive, cross-platform development tools for 3D video games, real-time 3D animation, and architectural visualization. Its editor runs on Mac OS X and Windows systems, and its creations can be published on Windows, Mac, and mobile platforms such as iPhone and Android and can be integrated into a web browser or player. The unique Unity 3D integrates integrated editing, graphics engine, resource import, one-click deployment, shaders, terrain editor, physics effects, audio, and video, and scripting to form a cascading, integrated development environment that creates high-quality 3D effects and realistic visuals. The cross-platform nature of Unity 3D is one of its most significant features and is the technology that drives the development of augmented reality-based experiential learning software [16].

Unity3D allows users to create simple geometric objects such as spheres, cubes, and rectangles and allows users to import models created by other 3D programs such as Maya, CATIA, and 3ds Max. Unity3D offers different types of licenses depending on the additional features; the basic version is free for individuals so that applications can be developed for private and commercial distribution. Unity3D also provides many functional modules for developers, including a global lighting system, a skeletal animation system, a script editor, particle, and environment effect editors.

(5) $$\begin{array}{c} M_{i}=\underset{j=1}{\sum }M_{ij}\left(\text{i}=1,2,3,\cdots ,n\right), \end{array}$$

(6) $$\begin{array}{c} E\left(k,j\right)={\left\|\left(R_{k}X^{j}+\pi t_{k}\right)\right\|}^{\sqrt{2}}. \end{array}$$

The basic development process can provide a base for the development of the curriculum unit. Detailed requirements analysis of the text unit is conducted based on the requirements analysis in the basic process design, including the analysis of the three-dimensional objectives and key points of the content of the unit, and the analysis of the characteristics of students learning the unit. Based on the structural design of the basic process, the detailed design of the course unit is completed, including instructional design and functional module design [17]. In the detailed design stage of the unit, the teaching design can design the learning situation, teaching content, teaching priorities, teaching process, and classroom control of the unit, while the design direction and content of the augmented reality teaching resources functional module of the unit are determined, and the methods and ideas in the design will be verified in the prototype production. After completing the detailed design of the unit, the accumulation of media materials is carried out according to the requirements of the objectives and functional module scripts, and the content of materials of high quality is collected as much as possible, including text, recognition pictures, augmented models, relevant audio, and video. After completing the preparation of materials, the augmented reality teaching resources of the unit are produced. Traditional computer-assisted teaching has gradually revealed its shortcomings in the wave of various new technologies. Augmented reality technology can effectively make up for the above shortcomings.

After the software project is built, it needs to be tested for deployment, operation, and performance, and then, the software is packaged for release. The software debugging stage mainly focuses on correcting various details of the software to present the best results when using it. Since the augmented reality presentation of the software is mainly through the recognition map to identify the real object, the operating environment is the user's operating range, and the recognition cards are divided according to different presentation contents, and one recognition card represents one presentation content, so during the debugging, corrections need to be made from the recognition map recognition effect, system content, positioning tracking, etc. The software is exported through the Unity 3D engine for packaging and distribution, first, select the “File” → “Build Settings” menu item in the Unity 3D navigation menu bar to open the “Build Setting” window and select the Android mobile platform for packaging and distribution.

## 4. AR Game Development and Implementation

Pronunciation teaching is crucial in teaching English to children. If a good pronunciation habit is not developed in children, it may cause long-term pronunciation errors, thus limiting the improvement of learners' overall English proficiency. There are two main difficulties in learning and correcting English pronunciation. On the one hand, bilingual learners tend to pronounce their mother tongue when learning a second language, for example, learners whose mother tongue is Cantonese tend to pronounce the “th” sound like the “f” sound, because this phenomenon is known as the negative effect of language transfer, which makes it difficult for learners to realize their pronunciation errors and makes it difficult for them to correct the pronunciation. On the other hand, there is a lack of professional native English-speaking teachers. According to statistics provided by the British Council, although there are approximately 1.5 billion English learners worldwide, only 250,000 native speakers are qualified to work as English teachers [18].

This case game is the research result of the author's team. The game is developed on the Android system, using 3ds Max and Magica Voxel modeling tools for the environment and character modeling and supported by the Mojang SDK development package provided by Storm Magic Mirror for the development and operation on the Unity 3D platform.

“Get To Know Your Phonetic Symbols Friends”, developed by the Institute, is a one-click English educational game based on virtual reality technology, in which learners are given the task of finding clues and making deductions based on details and the use of props. The learner enters the game and accepts the task of finding clues and reasoning, solving the corresponding questions, and finally succeeding in connecting the clues to get the reward of “research results”. The game flow is shown in Figure 2.

Through observation, it was found that students were slow to take off their headgear, exchanged words, and made loud noises when switching between the AR educational game learning activities and the teacher's lecture on the board. This phenomenon can be attributed to the “Game Transfer Phenomenon” in psychology, in which the players will recall the game music and game scenes in their brains after the game, and they cannot get out of the game for a long time. Therefore, I conducted a statistical survey on the time that learners switch to the real classroom in each game level, as shown in Figure 3, which shows that from the first to the last level of the game, students switching from virtual to real becomes a decreasing trend, and it shows a precipitous decrease after the first level and then tends to be stable.

Traditional English teaching in junior high schools often presents the content in programmed language. In terms of communication, students' stored information memory is often stolen in exchange for a smooth communication process. The teacher's repeated stimulation of knowledge points initially brings students a short period, and the teacher's monologue and students' responses are typical of the institutionalized mechanical process of “stimulus-response,” which later leads to a diminishing degree of students' response to knowledge [19]. The lack of the teacher's ability to grasp the rhythm of the scene, combined with the cognitive understanding that both teachers and students expect too much from the effect of online learning to a certain extent weakens the teaching effect of AR educational games. In other words, the use of AR educational games does not allow teachers to let go of the initiative in the classroom; rather, the use of technology causes student mood swings that require positive intervention by teachers.

Tracking accuracy is defined as the percentage of video frames where the distance between the center point of the target position estimated by the tracking algorithm and the center point of the manually labeled target position is less than a preset threshold. In general, the threshold value is defined as 20 pixel points. When the distance between the algorithm's estimated target position centroid and the actual target position point is less than the threshold pixel point, tracking fails. The same four tracking algorithms ESM, Inertial KLT, PhonyFerns, and ESM-SG-MB are used to test the accuracy of these two video frames, and the experimental results are shown in Figure 4, where the horizontal coordinates are the threshold pixels and the vertical coordinates are the tracking accuracy. The Internet has deeply influenced children since they began to receive education. They no longer stick to the small family around them but look at the whole world with curiosity. They are the most tempted individuals in the face of anything new.

As a psychological state that sustains and directs learners' behavior, the level of motivation governs learners' learning effectiveness. Malone, who was the first to begin research in this area, identified four elements that control motivation to play, namely, challenge, control, curiosity, and fantasy [20]. Positive emotions are the feelings of learners when they make progress in achieving their goals or when they are evaluated positively by the outside world, and how stimulating learners' positive emotions in the game context is the key to the success of AR educational games. Studies have found that users in the game will stimulate positive emotions through events such as point acquisition and goal achievement, and after these events are over, the arousal level will continue to drop exponentially [21]. The learning of language knowledge can never be separated from the specific context of use, and any language knowledge acquired from a single context must lack a structural level. In traditional English language teaching, students often acquire vocabulary and grammar knowledge that is not contextualized and presented in fragmented form, making it difficult for learners to transfer in face-to-face communication. In addition, learners lack confidence in their foreign language skills, and the greatest enemy of foreign language learners is the inexplicable feeling of anxiety. Compared with the actual language environment, it is easier for learners to let go of their guard and break their anxiety in the virtual space. In the AR environment, learners can choose their communication scenarios, objects, and difficulty levels and practice them repeatedly until they master them. It is undeniable that we all like entertainment and play games, and so do students. The relaxed atmosphere of games, full of exploration and fun, makes people want to play further. Based on this, educators try to introduce the mechanism of games into education. To stimulate students' interest to improve the atmosphere of the classroom.

Smartphones are the dominant platform for mobile augmented reality systems, which include inertial sensor devices such as accelerometers, gyroscopes, and magnetometers. While inexpensive sensor devices are often subject to noise during use that can skew the acquired data, we can still get a rough estimate of the device's orientation information from them. Android's software development kit provides application developers with functions that allow applications to use the device's sensors to obtain the device's orientation information. However, the smartphone is affected by electromagnetic fields in outdoor environments, resulting in significant jitter noise in the data measured by the accelerometer and magnetometer. As shown in Figure 5, the results obtained from the accelerometer and magnetometer of the smartphone in a smooth moving state and a state with a violent movement, respectively, are compared with the results filtered by the Kalman filter, with the horizontal axis representing the time and the vertical axis representing the angular change in the *x*-axis direction relative to the previously defined direction. As can be seen from the figure, jitter-free and drift-free direction values can be obtained using a simple compensation filter.

To evaluate the time metrics of the feature descriptors, 10 graphs with different feature points are selected here for testing. ORB, SIFT, SURF, and BRIEF are used for feature description and matching, respectively. To remove the effect of the time of feature detection, all feature descriptors are used here for feature extraction using the CenSurE method. The spatial complexity is defined as the maximum of the memory overhead required to run the process during the feature point description and matching. In this experiment, the five feature descriptors BRIEF, ORB, SIFT, SURF, and FREAK are compared, and the feature points are described and matched for the same image with a resolution of 480 × 640, and the memory consumption of the feature point detection phase is not considered here. The experimental results are shown in Figure 6. From Figure 6, we can see that the memory consumption of SIFT and SURF is large. Because SIFT uses 128-dimensional feature descriptors and floating-point type, it takes up 512 bytes of space. Similarly, SURF uses 64-dimensional feature descriptors, which also occupy 256 bytes of memory space. Therefore, SIFT and SURF consume a lot of memory when the image has many feature points. The descriptors such as BRIEF, ORB, and FREAK use binary code strings to match feature points with Hamming distance, so they consume less memory and are more suitable for mobile devices.

## 5. Analysis of the Application and Effectiveness of Children's English Pronunciation Teaching Based on AR Game Assistance

To better validate the effectiveness of the AR learning activities designed in this study, we conducted a week-long naturalistic observation of the classroom learning quality of the target students before the study began. In the three rounds of action research, we derived student scores for each round of action research by observing each student separately over time and then conducted paired-sample *t*-tests on the students' scores in the three rounds to observe the process of change in students' learning quality during the three rounds of action [22].

The assessment of pronunciation standards is based on KUDA's speech assessment function, and specific assessment contents are set in the assessment node. “The students' pronunciation standard was determined by comparing the standard pronunciation of the corpus with the pronunciation obtained from the system. In this study, the range of pronunciation standards was set from 0 to 10, as shown in Table 1, and the students in two classes were grouped into 8 groups of 10 students; the system would summarize the scores of each group and take the average, and finally, the weekly pronunciation standard scores were obtained, as shown in Figure 7.

In the first week, students were able to imitate the pronunciation given by the system in the follow-up activities, but the overall standard of pronunciation was low, and the lack of “completeness” of the sentences was an important factor in this result. As the learning activity progressed, the students received corrective and reinforcing feedback from the system, which led to a constant adjustment of their pronunciation norms [23]. The students' pronunciation level increased rapidly from the second week and reached a more stable level by the fifth week. The change curve of each student shows that the pronunciation standard of some students will decrease in the second week, mainly because of the active intervention and prompting of the teacher in the first week to avoid the students' loss of self-confidence, and this behavior starts to decrease gradually in the second week.

Based on the first and second rounds, it was found that students' speaking anxiety levels were mainly reflected in the size of their voices when answering questions, with louder voices indicating lower levels of anxiety and vice versa. The voice size judgment has different assessment criteria according to each student's habits. The specific method is that after all assessment sessions are finished, the system selects the maximum value from each student's weekly speaking voice and sets it to 100%, and all other voice sizes are compared with the maximum value and recorded in the form of a percentage, as shown in Figure 8.

According to the range of voice size distribution in the graph, the speaking anxiety level had a small decrease in the first three weeks, and then a more significant decrease in the fourth week, and tended to stabilize and approach the voice maximum in the fifth and sixth weeks [24]. Combined with the analysis of the classroom observation results, the students did not fully establish their sense of goal in the first week when they first started to encounter new knowledge, so they almost did not feel anxious, so the main reason for the low voice in the first week was that the students could not give feedback on the conversation content in time. The second week to the fourth week is the main time when students feel anxious and the stage of rapid proficiency in the learning content, until the fifth week when students' anxiety level starts to drop to the lowest, which is also the time when the target content is mastered.

At the end of the experiment, the most involved experimenters were given a questionnaire to measure their attitudes toward the learning environment. The questionnaire includes 3 dimensions software ease of use, software usefulness, and software satisfaction; each dimension contains 3 questions, a total of 9 questions; and the questionnaire is formed by setting a 5-level scale (1 means strongly oppose, 2 means oppose, 3 means neutral, 4 means agree, and 5 means strongly agree). The statistical results are shown in Figure 9.

As can be seen in Figure 9, the rating of the ease of use of the software (mean = 4.7112) is high, which shows that learners can easily operate access the AR educational game for learning. In other words, both teachers and students are looking forward to the next teaching experiment to enter their learning life, and this expectation not only urges the researcher to reform the English curriculum and teaching but also reflects that AR anticipation not only urges the researchers to reform the English curriculum and teaching but also reflects the fact that the application of AR in the classroom can increase students' motivation and participation [25]. In any case, the overall level of learners' attitudes toward the learning environment in the AR educational game was high, and most of the learners were positive about this learning method, and the software provided a better learning environment for the middle school classroom, and learners were able to maintain a high level of interest and initiative in learning. At the same time, the differences in attitudes toward AR educational games due to gender differences, which were feared before the experiment, did not show significant differences in the questionnaire.

## 6. Discussion

Pronunciation instructional standards are not sensory appealing to children, and complex and specialized pronunciation charts may be difficult for child learners to identify. Audio feedback is widely used in pronunciation instruction so that learners can understand pronunciation errors by comparing standard pronunciation with their pronunciation, but single audio feedback is also not sensorially appealing to children's learners. Audio feedback is not effective for children who have not yet mastered phonetic symbols. In offline pronunciation instruction, when learners have difficulty realizing their pronunciation errors, teachers make extensive use of oral pronunciation movement demonstrations, such as clear pronunciation (auditory), along with clear pronunciation movements (visual), to show how to pronounce the sounds correctly. For learners with serious pronunciation errors that are difficult to correct, teachers use more expressive and slightly exaggerated teaching methods to correct pronunciation: slowing down, exaggerating or dwelling on oral pronunciation movements (visual), and slowing down, repeating, or changing the pitch of speech (auditory) to reinforce the position of the incorrect pronunciation, helping learners to realize their pronunciation errors from the visual and auditory perspectives, respectively. Therefore, the image design of the virtual teacher with pedagogical expressiveness should adopt the appearance of children's favorite characters with distinctive colors and affinity. The image of the virtual teacher can be flat or three-dimensional or use novel AR or AR to display. The front angle needs to focus on the movement of the mouth, teeth, and tongue, and the side angle needs to focus on the movement of the important oral articulation organs (including the tongue, upper and lower lips, upper and lower teeth, jaw, and uvula). For children to understand the articulatory movements, the design of the articulatory organs needs to be simplified as much as possible.

Augmented reality technology, as an extension of virtual reality technology, brings people an unprecedented visual experience and makes them wonder at the infinite charm of modern technology. As a rapidly developing new form of software, it is constantly penetrating the field of learning and gradually promoting the development of the field of learning and research, bringing learners a wonderful experience in all aspects with its unique flexibility, practicality, and combination of reality and reality, and restoring the real sense of knowledge by building a seamless integration of virtual space and physical space and ubiquitous learning space, further satisfying the knowledge seekers' needs for interactivity. This study is based on a three-year study of augmented reality. After three years of tracking and exploring augmented reality, this study has achieved the span from model to entity and from theory to practice based on the research results and many mature products at home and abroad, and designed and developed augmented reality-based experiential teaching demonstration software. In the AR game children's English teaching, we also can not ignore the use of time, children's self-control if, a long-time uncontrolled use will make children indulge in it, ignoring the main purpose of learning, resulting in putting the cart before the horse.

## 7. Conclusion

Augmented reality, as a constantly developing and improving the technological tool, is gradually playing its unique role in the field of education. In this paper, we use mobile augmented reality technology as a teaching aid and practice and apply AR games to assist children's English pronunciation teaching. Based on the AR-based elementary school English experiential learning activity model, the case study is designed based on the elementary school English listening and speaking lesson “Get To Know Your Phonetic Symbols Friends.” In this case, the AR-based English learning software was designed and developed to support teaching and learning based on a needs analysis for the teaching experiment. The designed AR-based experiential learning activities were applied to the teaching practice and their effects were measured; data were collected through test papers, questionnaires, and interviews, and it was concluded that the AR-based experiential learning activities for elementary school English were recognized by students and teachers, and to a certain extent, they helped improve elementary school students' word learning ability and English conversation ability. It also has a positive impact on the improvement of learning interests. Due to the limitations of the author's personal ability and research conditions, this study still has the following shortcomings. The application of augmented reality in classroom teaching is still in the initial stage of exploration. Coupled with the limitations of time and experimental conditions, the sample cases and teaching contents selected in this study are few, so the experimental results obtained are not ruled out to be contingent. In the future, other course content will be added to further verify the experimental conclusions.

## Figures and Tables

**Figure 1:** AR educational game design framework.

**Figure 2:** “ Get To Know Your Phonetic Symbols Friends “ game tutorial.

**Figure 3:** Students' switching time curve between AR environment and real environment.

**Figure 4:** Comparison of algorithm accuracy.

**Figure 5:** Comparison of results of the model in different cases.

**Figure 6:** Memory consumption comparison results.

**Figure 7:** The change curve of pronunciation standard of students in each group.

**Figure 8:** Changes in student voice size.

**Figure 9:** Description of students' attitude towards learning environment for AR game teaching.

**Table 1:** Judgment standard of pronunciation standard.

Index	0-5	6-8	9-10
	Poor	Medium	Excellent
Completion		7	
Tone			9
Rhyme		6	
Fluency	5		
Loudness		8	

## Data Availability

The data that support the findings of this study are openly available at https://www.hindawi.com/journals/js/2021/2887302/ [doi:10.1155/2021/2887302], reference number [13].
